# Méningiome chordoïde extra-axiale: à propos d’un cas

**DOI:** 10.11604/pamj.2021.38.123.20437

**Published:** 2021-02-04

**Authors:** Mohammed Guini, Nabil Raouzi, Noureddine Oulali, Fayçal Moufid

**Affiliations:** 1 Service de Neurochirurgie, Centre Hospitalier Universitaire Mohammed VI, Oujda, Maroc

**Keywords:** Méningiome, chordoïde, Castelman, à propos d’un cas, Meningioma, chordoid, Castelman, case report

## Abstract

Une découverte fortuite d'une lésion de novo chez une patiente de 45 ans, la tomodensitométrie cérébrale réalisée montre une lésion ptérionale gauche intra-diploïque isodense avec une lyse osseuse, qui se rehausse de façon homogène après injection de produit de contraste, l'imagerie par résonnance magnétique montre une lésion hypointense en T1 et spontanément hyperintense en T2 FLAIR, et se rehausse très fortement après injection de Gadolinium. Une résection complète de la tumeur a été réalisée. Le diagnostic histologique était de méningiome chordoïde.

## Abstract (en)

This study reports the case of a 45-year-old female patient who underwent brain CT scan which fortuitously revealed de novo lesion. She was diagnosed with left isodense intradiploid lesion in the pterional region with bone lysis uniformly enhancing after injection of contrast medium. Magnetic resonance imaging showed T1-weighted hypointense lesion, spontaneously hyperintense signal on T2-weighted images and FLAIR images, strongly enhancing after gadolinium injection. Total tumor excision was performed. Histological examination showed chordoid meningioma.

## Introduction

Le méningiome chordoïde est un rare sous-type de méningiomes parfois associé à la maladie de Castelman [1], il représente entre 0.5 et 1% de tous les méningiomes [2-4], à cause de son haut potentiel de récidive, il a été classé parmi les méningiomes de grade 2 selon la dernière relecture de la classification des tumeurs du système nerveux établie par l´Organisation mondiale de la santé [5]. Le but de ce travail est d´étudier les caractéristiques cliniques et biologiques de cette entité et de discuter les principaux diagnostics différentiels.

## Patient et observation

Il s´agit d´une patiente âgée de 45 ans, qui a été victime d´un traumatisme crânien bénin suite à un accident de la voie publique, l´examen clinique était normal; notamment pas de signes méningés, ni de troubles de la sensibilité ou de la motricité. Le bilan biologique retrouve une anémie hypochrome microcytaire avec un taux d´hémoglobine à 8.1 g/dl mais sans syndrome inflammatoire. La tomodensitométrie puis l´imagerie par résonnance magnétique cérébrale retrouve une lésion extra-axiale intra-diploïque ptérionale gauche, avec une érosion de la structure osseuse, la lésion présentant un compartiment extra crânien de petite taille et une composante intracrânienne volumineuse, hypointense en T1 et se rehausse très fortement après injection de gadolinium, spontanément hyperintense en T2 et FLAIR, on note également que l´artère méningée moyenne gauche traverse la masse dans une partie de son trajet confirmant le caractère hypervasculaire de la lésion, cette dernière semblait être intra osseuse, sans envahissement du revêtement piale ni du cortex adjacent, avec un discret effet de masse (Figure 1, Figure 2), tous ces éléments on fait évoquer dans l´ordre un angiome intra-osseux, un hémangiopéricytome ou un méningiome hémangioblastique.

**Figure 1:** A) coupe axiale scanographique montrant une lésion extra-axiale ptérionale gauche associée à la présence de calcifications et avec un rehaussement intense et homogène après injection de produit de contraste iodé; B) fenêtre osseuse montrant une lyse de la table interne et discrète extension sous-cutanée par lyse de la table externe avec légère extension dans les parties molles de la fosse temporale externe gauche avec hyperostose péri lésionnelle

**Figure 2:** A) IRM coupe coronale T1 avec injection de gadolinium montrant une lésion expansive développée dans l'épaisseur du diploé au niveau de la région ptérionale gauche se rehaussant très fortement après injection gadolinium; B) la lésion est spontanément hyper-intense en FLAIR, sur cette coupe axiale on visualise le passage de l’artère méningée moyenne dans la masse tumorale, par ailleurs l´effet de masse est discret

**Intervention:** une artériographie crânio-faciale a été réalisée avant l´intervention montrant une vascularisation presque exclusive par des branches issues de l´artère méningée moyenne homolatérale, permettant une embolisation des artères nourricières principales. L´intervention chirurgicale menée par voie ptérionale gauche, retrouve mise à part l´ostéolyse une tumeur grisâtre gélatineuse et fibrineuse avec attache dure-mérienne obligeant à faire une incision circulaire à ce niveau permettant une exérèse Simpson grade 1.

L´examen anatomo-pathologique retrouve un tissu fibreux avec la présence de travées et de petits massifs de cellules physaliphores comportant un cytoplasme pâle éosinophile et des noyaux ovalaires sans atypie ni mitose manifeste, enchâssés dans une abondante substance mucoïde, infiltrant l´os et le muscle strié (Figure 3). Par ailleurs, on note la présence de plusieurs petits amas de prolifération de cellules d´aspect méningothéliales, constitués de lobules avec enroulement des cellules. L´étude immunohistochimique (IHC) effectuée montre la positivité des cellules pour la vimentine et l´antigène épithélial membranaire (EMA) et la négativité pour la cytokératine. Il s´y associe une intense positivité pour les anticorps anti-récepteurs de la progestérone, mais sans marquage pour les anticorps anti-récepteurs de l´œstrogène. Enfin, l´index de prolifération Ki67 (clone MIB 1) est inférieur à 1%. Le diagnostic retenu est celui de méningiome chordoïde.

**Figure 3:** A) composante méningothéliale (lobules des cellules fusiformes avec enroulement) et chordoïde (travées et amas de petites cellules au cytoplasme éosinophile); B) bleu alcian montrant le fond mucoïde entourant des massifs de petites cellules (composante chordoïde); C) positivité de l'EMA des deux composantes cellulaires; D) négativité de la cytokératine AE1/AE3

**Evolution:** la patiente, revue à 10 jours puis à un mois puis à trois mois de l´intervention, présente un examen clinique normal et un bilan biologique sans particularité, notamment pas d´anémie à la numération formule sanguine. L´IRM de contrôle montre une exérèse complète de la tumeur sans prise de contraste méningée ni œdème cérébrale.

## Discussion

Les méningiomes chordoïdes ont été décrits pour la première fois par Kepes *et al*. en 1988, comme étant une tumeur qui se présente préférentiellement chez les enfants, et souvent associé à la maladie de Castelman [1]. Depuis notre compréhension de cette tumeur a considérablement augmentée; l´incidence estimée est de 0.5 à 1% des méningiomes traités chirurgicalement avec une légère prédominance féminine [4-6]. Les symptômes révélateurs diffèrent selon la localisation et la taille mais le symptôme le plus fréquent reste les céphalées, sans aucun signe spécifique objectif retrouvé dans la littérature des méningiomes chordoïdes [1,2,4,7,8]. La maladie de Castleman ou l´hyperplasie ganglionnaire angiofolliculaire, décrite pour la première fois en 1956 par Benjamin Castleman [9,10], est une maladie lymphoproliférative rare, typiquement sous forme des masses médiastinales ou hilaires hypervasculaires. Elle se révèle soit par un syndrome tumoral lié à la compression d´organes de voisinage, soit par un syndrome inflammatoire systémique avec hyperthermie, sueurs nocturnes et altération de l´état général, associé à une hypergammaglobulinémie. Kepes *et al*. [1] décrit sept jeunes patients présentant un méningiome chordoïde associé à quelques signes de la maladie de castelman, notamment deux patients dont l´anémie hypochrome microcytaire, résolutive immédiatement après l´exérèse macroscopiquement complète de la tumeur, est réapparue avec la récidive locale de cette tumeur.

Cependant, Couce *et al*. [4] ne rapporte aucun cas d´anémie ou dysglobulinémie parmi les 42 cas de méningiomes chordoïdes chez l´adulte; ZHU Hong-da *et al*. [11] a colligé 17 cas de méningiomes chordoïdes et dont 3 patients présentaient une anémie hypochrome microcytaire sans autre signes associés, notre cas présente également le même tableau, d´autres auteurs [4-8] ont constaté que l´infiltration lymphoplasmocytaire péritumorale d´un méningiome choroïde est prédominé par les lymphocytes B chez les jeunes patients alors que chez les patients adultes. Il existe une prédominance des lymphocytes T, Kaloshi *et al*. [12] pour sa part pense que l´expression tumorale de l´interleukine 6 pourrait expliquer les manifestations systémiques de la maladie de Castelman, et que la disparition des symptômes systémiques après une exérèse complète de la tumeur appuis son hypothèse (Tableau 1).

**Tableau 1:** comparaison de données clinicopathologiques observées chez plusieurs séries de méningiomes chordoïdes

Données épidémiologique	Informations générales				Localisation tumorale		Manifestations systémiques		Pourcentage des éléments chordoïdes		Suivi	
	Nombre de cas	l'Age moyen	Nombre d'enfants moins de 18 ans	Sex ratio	Supra-tentorielle	Infra-tentorielle	Typique	Atypique	>50%	<50%	Radio-thérapie	Taux de récidive
Kepes *et al*.	7	8-19 (11,9)	6 (85,7%)	1:1,3	71,4%	28,6%	100%	-	-	-	-	28,6%
Epari *et al*.	12	12-67 (32,4)	3 (25%)	1:1,4	66,7%	33,3%	100%	-	91,6%	8,3%		0%
Lin *et al*.	11	43-77 (60,8)	-	1,2:1	91%	9%	-	100%	69%	31%	27%	20%
Couce *et al*.	42	12-77 (47.4)	12-77 (47.4)	1:1,1	88%	12%	88%	12%	81%	19%	-	42%
X-Q Wang *et al*.	30	16-74 (49,6)	1 (5,8%)	1:1,3	80%	20%	0%	100%	69%	31%	30%	19%

La confirmation diagnostic du méningiome chordoïde est histopathologique, il s´agit d´une prolifération de cellules tumorales épithélioïdes ou fusiforme agencée en travées et cordons, comportant un cytoplasme pâle et éosinophile avec des noyaux ovalaire et dense, baignant dans une trame mucoïde abondante, avec expression à l´immunohistochimie de l´EMA et la vimentine, et négativité de la cytokératine ce qui la différentie du chordome: le diagnostic différentiel principale à côté du gliome chordoïde qui exprime de façon intense la GFAP (Glial Fibrillary Acid Protein) [13], il existe d´autres diagnostics différentiels: ce sont des tumeurs avec cytoplasme pâle, une structure mucoïde/choroïde et qui peuvent se développer dans et/ou proche du système nerveux centrale telle que: le chordome chordoïdes, chondrosarcome myxoïde, chondrosarcome de bas grade, enchondrome, carcinome métastatique mucineux et le carcinome métastatique de cellules rénale [3].

L´exérèse chirurgicale reste le traitement de choix et le résultat désiré sera une exérèse macroscopiquement totale, vu le haut potentiel de récidive de ce type de méningiome le classant au grade 2 de la classification de l´OMS, malgré l´absence des critères de malignité (index mitotique élevé, nécrose, envahissement cérébral), sauf que, dans des cas de méningiomes, telle que ceux envahissant le sinus caverneux, la région petroclivale, la partie postérieure du sinus sagittale supérieure, ou le nerf optique, l´exérèse totale est impossible vu le risque vitale ou par rapport aux structures vasculaires [14], dans ce genre de situations une exérèse subtotale suivie d´une radiothérapie adjuvante ou une radiochirurgie stéréotactique est recommandé surtout quand le méningiome est de grade 2 ou 3 de l´OMS [3].

## Conclusion

Le méningiome chordoïde est une tumeur particulière, même si les différentes séries ne trouvent pas toujours une association avec la maladie de Castelman, ni une préférence d´âge, c´est une tumeur redoutable de récidive et dont le diagnostic est basé sur l´étude immunohistochimique.

## References

[1] Kepes JJ, Chen WY, Connors MH, Vogel FS (1988). "Chordoid" meningeal tumors in young individuals with peritumoral lympho plasma cellular infiltrates causing systemic manifestations of the Castleman syndrome: a report of seven cases. Cancer.

[2] Epari S, Sharma MC, Sarkar C, Garg A, Gupta A, Mehta VS (2006). Chordoid meningioma, an uncommon variant of meningioma: a clinicopathologic study of 12 cases. J Neurooncol.

[3] Lin JW, Ho JT, Lin YJ, Wu YT (2010). Chordoid meningioma: a clinicopathologic study of 11 cases at a single institution. J Neurooncol.

[4] Couce ME, Aker FV, Scheithauer BW (2000). Chordoid meningioma: a clinicopathologic study of 42 cases. Am J Surg Pathol.

[5] Louis DN, Perry A, Reifenberger G, von Deimling A, Figarella-Branger D, Cavenee WK (2016). The 2016 World Health Organization classification of tumors of the central nervous system: a summary. Acta Neuropathol.

[6] Tena-Suck ML, Collado-OrtÃ¬z MA, Salinas-Lara C, García-López R, Gelista N, Rembao-Bojorquez D (2010). Chordoid meningioma: a report of ten cases. J Neurooncol.

[7] Mitsuhashi T, Ono S, Inohara T, Otomo T, Aoki A, Ueki Y (2006). Chordoid meningioma: case report. Neurol Med Chir (Tokyo).

[8] Wang XQ, Mei GH, Zhao L, Li ST, Gong Y, Zhong J (2013). Clinical features and treatment of intracranial chordoid meningioma: a report of 30 cases. Histopathology.

[9] Castleman B, Towne VW (1954). Case records of the Massachusetts General Hospital: case 40231 (hyperplasia of mediastinal lymph nodes). N Engl J Med.

[10] Castleman B, Iverson L, Menendez VP (1956). Localized mediastinal lymph node hyperplasia resembling thymoma. Cancer.

[11] Zhu HD, Xie Q, Gong Y, Mao Y, Zhong P, Che XM (2013). Chordoid meningioma: a retrospective study of 17 cases at a single institution. Chin Med J (Engl).

[12] Kaloshi G, Vreto G, Lame A, Kerri I, Bushati T, Rroji A (2011). Report of two cases of chordoid meningioma in patients with Castleman syndrome. J Neurooncol.

[13] Cho HY, Lee M, Takei H, Dancer J, Ro JY, Zhai QJ (2009). Immunohistochemical comparison of chordoma with chondrosarcoma, myxopapillary ependymoma and chordoid meningioma. Appl Immunohistochem Mol Morphol.

[14] Whittle IR, Smith C, Navoo P, Collie D (2004). Meningiomas. Lancet.

